The article "Lifestyles of Spanish elders from supervened SARS-CoV-2 variant onwards: A correlational research on life satisfaction and social-relational praxes" was published in 2022. Journal: Front Psychol.

# Lifestyles of Spanish elders from supervened SARS-CoV-2 variant onwards: A correlational research on life satisfaction and social-relational praxes

**DOI:** 10.3389/fpsyg.2022.948745

**Published:** 2022-09-28

**Authors:** Orlanda Díaz-García, Inmaculada Herranz Aguayo, Patricia Fernández de Castro, José Luis Gómez Ramos

**Affiliations:** ^1^Department of Labour Law and Social Work, Faculty of Social Sciences of Talavera de la Reina, University of Castilla-La Mancha, Ciudad Real, Spain; ^2^Department of Philosophy, Anthropology and Sociology, Faculty of Social Sciences of Talavera de la Reina, University of Castilla-La Mancha, Ciudad Real, Spain; ^3^Pedagogy Department, Faculty of Education at Albacete, University of Castilla-La Mancha, Ciudad Real, Spain

**Keywords:** elderliness, lifestyles, satisfactoriness, leisureliness, resocialization

## Abstract

**Objective:**

This study aimed to analyze the influence and measurement of the relationship and interaction between the elderly lifestyles after the appearance of the SARS-CoV-2 variant and the factors analyzed comprised life satisfaction levels, social relationships, and daily-life activities.

**Methods:**

The study population was ≥ 65 in Castile-La Mancha (*N* = 390,221). The research design was quantitative and arose from primary data collected via an ad hoc survey carried out through the Computer Assisted Telephone Interview system by randomly stratified sampling. The sample size was made up of 1,065 cases, and the participants were selected through a random sampling stratified by gender quotas (55.40% women; 44.60% men), age ($\bar{x}\;=\;76.56$), province, and habitat size.

**Results:**

The results obtained revealed two main lifestyles, from which a notable behavioral change in personal relationships led to infer toward alternative lifestyles.

**Conclusion:**

Notwithstanding the variation in lifestyles of the elderly after the pandemic, certain relationships remained unaltered. Thus, from the analyzed variables, relatives and friends relationships were scarcely influenced by the supervened incident.

## Introduction

The aging of the population is yet a consolidated trend worldwide, having been estimated that the number of older adults will increase considerably around the world in the nearest future, being even presumed to double by 2050 (United Nations, 2019). In this regard, the population aged 65 and over comprised 19.43% of the total inhabitants in Spain in 2020 (Instituto Nacional de Estadística, 2020), with an increasing rate of migrants (Ciobanu et al., 2017). The boundary of ≥ 65-year-olds is set in this study because it is the current official age in Spain at which citizens' retirement starts. Thus, this transition from professional activity to leisureliness is associated with significant social, economic, and relational changes in people's lives. Apropos of such a trend, the Instituto Nacional de Estadística (2020) estimates that this age range faction will reach 31.44% by 2050. The global aging-raising trend has also favored the rapid increase of research on discovering the factors influencing optimal aging revealed through lifestyles in humankind. To Rowe and Kahn (1997), successful aging comprises the absence of disease, the preservation of functional skills, and the ongoing commitment to life, all interrelated factors toward achieving pleasant aging leading to specific activities (Rowe and Kahn, 1997; Herranz et al., 2013; Bulow and Söderqvist, 2014; Urtamo et al., 2019).

The article "Lifestyles of Spanish elders from supervened SARS-CoV-2 variant onwards: A correlational research on life satisfaction and social-relational praxes" was published in 2022. Journal: Front Psychol.

Due to migration facts and that “[t]here will be two billion people in old age category worldwide by 2050” (Pant and Subedi, 2020, p. 32), not only does pleasant aging needs to be linked to pleasing-physical wellbeing but also does the *idiosyncrasy* and the sense of living a meaningful life (VanderWeele, 2017; Steptoe and Fancourt, 2019). If we ponder the term from a heterogeneous perspective, satisfactory livingness remains the most common concept in the literature to measure the subjective wellbeing of the superannuated (Fagerström et al., 2007; Ju, 2017; Tomioka et al., 2017; Etxeberría et al., 2019; Steptoe and Fancourt, 2019). Thus, to spot how the ab ovo stay-at-home to prevent further spreading of SARS-CoV-2 influenced lifestyles, we analyzed the concept of successful aging from the type and frequency of daily activities carried out by people aged 65 and above. Congruously, this investigation also adopts a social perspective and acknowledges the social relationships established by the analyzed sample with their homonyms and heteronyms.

### The myth of elderly's lifestyles

Just as the lifestyles established from interpersonal relationships are linked to the type and frequency of daily life and the activities carried out by people (Geithner and Wagner, 2022), the dimension of life satisfaction (i.e., economic situation; sexual/affective relations; health; leisure, appearance, personal abilities; family, friends, or colleagues; spare time) is mirrored in the multiple aspects of social life and the distinct areas of personal joy (Fagerström et al., 2007; Von Humboldt and Leal, 2017; Gumà and Arpino, 2021). From the empirical evidence about the connection between lifestyles and satisfaction with life, it is observed that the higher the satisfaction with life, the more the other positive life aspects increase and vice versa (Toepoel, 2013; Gutiérrez et al., 2014; Vozikaki et al., 2017). Indeed, incomes also influence lifestyles, social-relational praxes, and behaviors (Xue et al., 2021).

The article "Lifestyles of Spanish elders from supervened SARS-CoV-2 variant onwards: A correlational research on life satisfaction and social-relational praxes" was published in 2022. Journal: Front Psychol.

An example of the above can be observed in Gumà and Arpino's (2021) research, where participants' satisfaction with life is more significant when their occupational contribution (domestic or professional) increases. To these authors, such satisfaction levels become more notable when *wealthiness* and *healthiness* concur. Other factors influencing the significant relationships among life-satisfied elders are those linked to the yet mentioned health, financial situation, family, and social contacts or relationships (Fagerström et al., 2007; Schnettler et al., 2014; de Albuquerque Araújo et al., 2020; Zadworna, 2022). To Pérez-Escoda (2013), when a correlation is established between the different aspects of people's satisfaction with life (family, health, work, and personal relationships), a determined quantitative weight is established for each bounding aspect.

Yet, not only the significant correlational relationship between the different aspects of life satisfaction in elderliness have been studied but such factors are also primarily studied from those perspectives associated with lifestyles and personal relationships (Molero and Pérez-Fuentes, 2011; Sampaio and Ito, 2013; Marques et al., 2016; Von Humboldt and Leal, 2017; Han et al., 2022; Penton et al., 2022), as much as from the perspective of indoor and outdoor activities (Silverstein and Parker, 2002; Triadó et al., 2009; Lee et al., 2014; Aponte, 2015; Santaella and Bohórquez, 2017; Vozikaki et al., 2017; Li et al., 2021; Chen et al., 2022; Geithner and Wagner, 2022). Similarly, the effect of personal relationships, particularly with family and friends, on life satisfaction is widely documented (Cornwell et al., 2008; Cheng et al., 2009; Litwin and Shiovitz-Ezra, 2011; Rafnsson et al., 2015; Burholt et al., 2020; LaBorde and Williams, 2022). From the literature, another aspect worth to be mentioned is that adults get higher satisfaction from life as they have more relatives than friends (Tomini et al., 2016).

## Materials and methods

The research goal consists of analyzing the influence and the relational and interactional connections between the three dimensions studied and considered fundamental in the lifestyle scrutiny of 65-year-olds onwards in the Autonomous Region of Castile-La Mancha, Spain. To say, *satisfaction levels* (D_1), *social relationships* (D_2), and *daily living activities* (D_3). From the referenced goal, a dyad of objectives emerges for the in-depth exploration of the grouped variables within each of the dimensions concerning the correlational analysis (O_1) and the enquiring on the influence and the interaction of groups between the levels of satisfaction, the frequencies in the social relations, and the frequency of activities as variables might have been originating different lifestyles (O_2).

The article "Lifestyles of Spanish elders from supervened SARS-CoV-2 variant onwards: A correlational research on life satisfaction and social-relational praxes" was published in 2022. Journal: Front Psychol.

### Instruments

The instrument for data collection is an ad hoc questionnaire implemented as a survey on a Spanish sample (Table 1). The duration of the research lasted 5 months (January to May 2021). The main categories and dimensions of the questionnaire, which are related to the objectives of this study, were the following: profile and sociodemographic variables (CD_1); living conditions (CD_2); household structure (CD_3); life habits (CD_4); socioeconomic indicators (CD_5); health and impact of the COVID-19 pandemic (CD_6); dependency and disability (CD_7); use of time (CD_8); leisure and culture (CD_9); use of information and communication technologies (CD_10); physical activity (CD_11); values and attitudes (CD_12); expectations and interests (CD_13); and perception and use of specialized services (CD_14).

**Table 1:** Data sheet.

Location	Castile-La Mancha, Spain
Population	≥65-year-olds (*N* = 390,221 [to date January 1, 2020])
Methodology	Computer Assisted Telephone Interviewing (CATI) survey
Sample size	*n* = 1,065 individuals/cases from the target population
Confidence interval	95%
Margin of error for the estimate	3%
Sampling distribution and quotas	Proportional sampling distribution by provinces. Representative survey process, stratified by sex quotas, age group, and habitat size
Fieldwork schedule	From January 5 to January 22, 2021
Questionnaire preparation time	15 min

Thus, because of its proximity to research goals, the results presented in this study constitute the analysis of just three of the dimensions contemplated from the full version of the questionnaire: *life satisfaction levels* (D_1); *interpersonal relationships* (D_2); and *type and frequency of day-to-day activities* (D_3). The dimensional components are detailed as follows:

#### D_1: Satisfaction with different aspects of life

This dimension is measured using gradual scales one-to-four whose values are revealed as follows: 1 = Not satisfied at all; 2 = Not very satisfied; 3 = Fairly satisfied; 4 = Very satisfied; and 98 = Not applicable. The factors measured in this item correspond to family, friends, neighbors, colleagues (residence, cultural center, social center, etc.), professional environments (gym, day center, library, and health center), sexual/affective relationships, health, physical, and cognitive abilities, appearance or personal image, financial situation, and leisure and free time. The questionnaire is widened from the scale of satisfaction with different aspects of life provided by Centro de Investigaciones Sociológicas. (2020a), as well as on the Effects and Consequences of COVID-19 scale (Centro de Investigaciones Sociológicas., 2020b,c). It also encompasses items from the Study on Public Opinion and Fiscal Policy held between 2010 and 2017 (Centro de Investigaciones Sociológicas., 2020d) and the Study 3201 parallel carried out by the Spanish General Social Survey (SGSS [in Centro de Investigaciones Sociológicas., 2018]).

The article "Lifestyles of Spanish elders from supervened SARS-CoV-2 variant onwards: A correlational research on life satisfaction and social-relational praxes" was published in 2022. Journal: Front Psychol.

#### D_2: Interpersonal relationships

This dimension is measured using a 1–4 personal contact frequency scale: 1 = Every day or almost every day; 2 = At least one time a week; 3 = At least one time a month; 4 = At least one time a year; and 98 = Not applicable. The personal relationships enquired about referred to a fellow club or association members; the number of offspring not living in the same locality; the number of offspring living in the same locality but not with the interviewee; grandchildren, siblings, cousins, and other relatives; friends who are not neighbors; neighbors; others; and caregivers (type of personal contact post-coded from the others). The scale is adapted from the frequency of contact in relationships (Centro de Investigaciones Sociológicas e Instituto de Migraciones y Servicios Sociales, 1998) and the frequency of carrying out activities with different people (Centro de Investigaciones Sociológicas e Instituto de Migraciones y Servicios Sociales, 1998).

#### D_3: Daily life and activities carried out and their frequency

To explore this dimension, the information is collected through two enquiries: the first on social and leisure activities (D_3.1) and the second on the frequency of activities carried out (D_3.2). The activity frequency scale keeps patterns like the previous ones (1–4 scales) whose values were as follows: 1 = Every day or almost every day; 2 = At least one time a week; 3 = At least one time a month; and 4 = At least one time a year. The scale is adapted from Attendance to Cultural and Leisure Activities and Activities of a Social Nature (Instituto Nacional de Estadística, 2011). The set of activities on which information has been extracted is 23, where some of the examples refer to visiting and receiving visitors (at home [including eating or having coffee together]); eating or dining away from home with family or friends; getting together to play cards or other games; going for tapas, drinks, having an aperitif, having a coffee, beer, or wine at a bar or a coffee shop; going dancing (orchestral dances, discos, lounge); attending a course, workshop, or seminar; attending conferences, gatherings, or discussion forums; going to the movies; going to the theater, ballet, concerts, and magic shows.

The article "Lifestyles of Spanish elders from supervened SARS-CoV-2 variant onwards: A correlational research on life satisfaction and social-relational praxes" was published in 2022. Journal: Front Psychol.

### Analysis procedure

To present the main descriptive results on each of the analyzed dimensions displayed in the previous epigraph, the choice of the fitting model's central tendency (*M*) measure is chosen to subsequently proceed to the correlational analysis (*p* < 0.01). This correlational research is performed via Pearson's correlation coefficient (intra- and inter-dimensional). The enquiry about the consistency and the explanatory weight of the analyzed dimensions on the social relations is carried out employing the linear multiple regression analysis.

## Results

Research results can be identified in two extensive blocks. The first segment (a) represents the interpretation of each dimension (satisfaction levels, social relationships, and activities of daily life), all linked to the correlations between the different aspects analyzed in each dimension to determine the main internal groupings revealed. The second segment (b), which is the aim of this study, explores the interactional relationship between the dimensions and the power or strength between the variables.

### Lifestyles: Satisfaction levels, social relationships, activities, and daily life

The satisfaction levels with the different aspects of life (D_1) are formed as self-perception indicators about people's lifestyles and vital situations. Thus, when averaging data, the results revealed that (inter)personal relationships are the aspects providing the analyzed population higher satisfaction levels (family [$\bar{x}=3.51$], friends [$\bar{x}=3.22$], professionals [$\bar{x}=3.10$], colleagues [$\bar{x}=3.01$], and neighbors [$\bar{x}=3.00$]). Contrarily, among the surveyed, the least valued aspects of life were those associated with the monetary state, sexual or affective relations, and health state (Figure 1).

**Figure 1:** Averaged satisfaction levels with the different aspects of life.

Personal relationships are constituted as the aspects that generate the most remarkable satisfaction levels; satisfaction with family and friends also maintains a robust correlation with the rest of the factors analyzed (*p* < 0.01). Consequently, the high satisfaction levels with family and friends coincide with the different aspects analyzed (Table 2).

**Table 2:** Interpersonal and intrapersonal satisfaction levels.

		**Satisfaction levels with**											
		**I**	**ii**	**iii**	**iv**	**v**	**vi**	**vii**	**viii**	**ix**	**x**	**xi**	**xii**
Satisfaction levels with family	(1)	1	0.490^**^	0.309^**^	0.243^**^	0.282^**^	0.184^**^	0.250^**^	0.227^**^	0.111^**^	0.146^**^	0.198^**^	0.192^**^
	(2)	–	0.000	0.000	0.000	0.000	0.000	0.000	0.000	0.000	0.000	0.000	0.000
	(3)	1,062	1,055	1,024	747	862	695	1,059	1,057	1,056	1,037	1,058	1,048
Satisfaction levels with friends	(1)	0.490^**^	1	0.511^**^	0.421^**^	0.351^**^	0.261^**^	0.277^**^	0.282^**^	0.193^**^	0.163^**^	0.236^**^	0.284^**^
	(2)	0.000	–	0.000	0.000	0.000	0.000	0.000	0.000	0.000	0.000	0.000	0.000
	(3)	1,055	1,056	1,018	745	858	691	1,053	1,051	1,050	1,031	1,052	1,043

(i) Family; (ii) Friends; (iii) Neighbors; (iv) Partners; (v) Professionals; (vi) Sexual/affective relations; (vii) Health; (viii) Skills; (ix) Self-image; (x) Financial situation; (xi) Free time; (xii) Leisure. (1) Pearson correlation, (2) Sig. (Bilateral), and (3) Bold represent the strongest relationships between variables.

** marks that the correlation is significant at the 0.01 level.

The article "Lifestyles of Spanish elders from supervened SARS-CoV-2 variant onwards: A correlational research on life satisfaction and social-relational praxes" was published in 2022. Journal: Front Psychol.

Having shown the high satisfaction levels prompted by the social interactions, the frequency of contact between the different groups is exposed (D_2). Regarding the frequency of social relationships, family relationships are the most assiduous (children in the same locality but not living together = 55.2%; grandchildren = 37.9%; children outside the locality = 28.6%). In the case of non-family social relationships, the frequency of contact is 46.7% in friends and 44.8% in neighbors. All the variables that affect personal contacts correlate significantly with each other.

Two differentiated relationships emerge from the analysis when observing the strongest correlations between variables. On the one hand, there are different family relationships with each other (“offspring living in the same locality” correlates with the “frequency of contact with offspring living outside city boundaries” [*r* = 0.643] and with “grandchildren” [*r* = 0.622]). On the other hand, there are established relationships between non-family contacts on both the “frequency of contact with friends” and “frequency of contact with neighbors (AmE)” [*r* = 0.448]).

The variables that affect the relationship with different personal contacts correlate significantly between them so that those who maintain frequent contact with one of the groups of people also maintain it with others and vice versa. However, if we stop at the most robust correlations, two distinct relationships reappear. Family relationships maintain a strong correlation among them both (“offspring living in the same locality” correlates with the frequency of contact with “offspring living outside city boundaries” [*r* = 0.643] and with “grandchildren” [*r* = 0.622]). Meanwhile, non-family relationships and friends and neighbors present the highest correlations between themselves (*r* = 0.448).

The article "Lifestyles of Spanish elders from supervened SARS-CoV-2 variant onwards: A correlational research on life satisfaction and social-relational praxes" was published in 2022. Journal: Front Psychol.

The third dimension of analysis (D_3) refers to the performance and frequency of the sets of daily activities (Table 3). If we focus on carrying out activities in the daily life of people over 65 in Castile-La Mancha, the most common activities are “talking on the phone with family and friends,” “walking” (accompanied), “eating or dining out,” and “visiting and entertainment.” However, not all activities are carried out with the same frequency. Among them all, a higher percentage of activities carried out every, or almost every, day is “talking on the phone with family and friends” (82%) and “going for a walk” (77.7%).

**Table 3:** Daily activities from the age of 65-year-old and above.

Visit and receive visits	55.8%
Eating or dining out home	58.4%
Going for a walk (accompanied)	73.7%^*^
Talking on the phone with family and friends	74.6%^*^

* Every day or almost every day.

Again, the correlation analysis between the performance frequencies of the different activities reveals two differentiated groups (Table 4). On the one hand, strong correlations were observed between the variables that show a high level of activity and diversity in leisure time outside the home and are the most linked to consumerism (*p* < 0.01). Contrarily, activities of a more traditional nature were linked to lower activity levels and social interactions.

**Table 4:** Correlation on activity performance.

		**Frequency levels with**												
		**I**	**ii**	**iii**	**iv**	**v**	**vi**	**vii**	**viii**	**ix**	**x**	**xi**	**xii**	**xiii**
Frequency level on visiting and receiving visits	(1)	–	0.241^**^	0.381^**^	–	–	0.238^**^	–	–	0.427^**^	0.448^*^	–	–	–
	(2)	–	0.000	0.000	–	–	0.000	–	–	0.000	0.011	–	–	–
	(3)	–	423	286	–	–	490	–	–	189	31	–	–	–
Frequency level on eating or dining out at home	(1)	0.241^**^	–	0.461^**^	0.569^**^	0.187^**^	0.244^**^	0.308^**^	0.353^**^	–	–	0.251^**^	0.433^**^	0.268^**^
	(2)	0.000	–	0.000	0.000	0.000	0.000	0.002	0.001	–	–	0.000	0.004	0.000
	(3)	423	–	371	50	518	516	100	79	–	–	323	43	339

(i) Visiting and receiving visits; (ii) Have lunch or dinner off home; (iii) Go for tapas, drinks, and aperitifs; (iv) Go dancing; (v) Go for a walk (accompanied); (vi) Talk on the phone with family and friends; (vii) Go to the movies; (viii) Go to the theater, ballet, and concerts; (ix) Go to church or religious activities; (x) Go to folkloric, bullfighting, and sports shows; (xi) Go to shopping centers; (xii) Go to the library or rearing club; (xiii) Read books, newspapers, and magazines. (1) Pearson correlation, (2) Sig. (Bilateral), and (3) Bold represent the strongest relationships between variables.

* marks that the correlation is significant at the 0.05 level

and

** marks that the correlation is significant at the 0.01 level.

The article "Lifestyles of Spanish elders from supervened SARS-CoV-2 variant onwards: A correlational research on life satisfaction and social-relational praxes" was published in 2022. Journal: Front Psychol.

Two large groups are observed from analyzing the main correlations within each dimension. In the dimension “satisfaction with different aspects of life” (D_1), we found a group of significant correlations (*p* < 0.01). Such correlations between family relationships and satisfaction levels in non-family relationships (friends and neighbors) concur. In the case of the dimension that measures the frequency in social relationships (D_2), we also found two groups of significant correlations (*p* < 0.01). On the one hand, the different family relations (children and grandchildren) are observed; on the other hand, non-family relationships (friends and neighbors) are revealed. Such correlations would indicate that, in cases in which there is a high frequency of contact with children, it also occurs in other family relationships. Similarly, when there is a high frequency of contact with friends, there is also a contact frequency in other relationships that are not family. Such results reveal a certain continuity with the results of D_1.

Finally, the correlations between the frequency of performing the group of activities of daily life (D_3.2) have also been analyzed, from which two different groups emerge between (I) the activities most linked to leisure and outside home activities and consumerism; and (II) the more traditional activities implying higher levels of inactivity or sedentariness. After the pandemic, such dimensional dualities might have justified the interactional analysis between the three proposed dimensions on the relationships between elderly groups and their lifestyles.

### Interaction between dimensions

The following subsections show (i) the interaction between satisfaction levels and contact frequencies and (ii) the frequency of activities and social relationships to show how the groupings presented above provide continuity to the relationship between the dimensions.

#### Satisfaction levels and frequency of contacts

When connecting respondents' satisfaction levels (D_1) with the frequency of contact in their social relationships (D_2), their frequency of contact with people increases and so does their satisfaction levels with the different aspects evaluated (*p* < 0.01). Also, it was observed that the contact frequency with relatives (offspring/grandchildren living in the same locality) establishes significant correlations with the rest of satisfaction levels: family, friends, neighbors, colleagues, professionals, etc. (Table 5). This correlation is inverse when it concerns the “level of economic satisfaction.” That is, in all cases, the greater the relationship with “offspring or grandchildren living in the same locality,” the lower the satisfaction level with their “financial situation.”

The article "Lifestyles of Spanish elders from supervened SARS-CoV-2 variant onwards: A correlational research on life satisfaction and social-relational praxes" was published in 2022. Journal: Front Psychol.

**Table 5:** Correlations between frequency of socio-family contact and satisfaction levels.

		**Frequency of contact with**		**Satisfaction levels with**					
		**i**	**ii**	**iii**	**iv**	**v**	**vi**	**vii**	**viii**
Frequency of contact with offspring living in the same city	(1)	1	0.622^**^	−0.335^**^	−0.284^**^	−0.166^**^	−0.171^**^	−0.217^**^	0.097^**^
	(2)	–	0.000	0.000	0.000	0.000	0.000	0.000	0.004
	(3)	924	838	924	919	894	660	758	900
Frequency of contact with grandchildren	(1)	0.622^**^	1	−0.259^**^	−0.229^**^	−0.204^**^	−0.202^**^	−0.166^**^	0.117^**^
	(2)	0.000	–	0.000	0.000	0.000	0.000	0.000	0.001
	(3)	838	881	881	875	855	619	718	857

(i) Offspring living in the same city; (ii) Grandchildren; (iii) Family; (iv) Friends; (v) Neighbors; (vi) Partners; (vii) Professionals; (viii) economic status. (1) Pearson correlation. (2) Sig. (Bilateral). (3) Bold represent the strongest relationships between variables.

** marks that the correlation is significant at the 0.01 level.

When analyzing and comparing the set of significant correlations (*p* < 0.01) with the “frequency of contact with friends,” the most robust correlations emerge from the levels of satisfaction with non-family personal relationships: friends, neighbors, colleagues, and professionals (Table 6).

**Table 6:** Satisfaction levels from non-family interrelations.

		**Satisfaction levels with**					
		**i**	**ii**	**iii**	**iv**	**v**	**vi**
Satisfaction levels with friends	(1)	1	−0.065^*^	−0.207^**^	−0.145^**^	−0.150^**^	−0.179^**^
	(2)	–	0.037	0.000	0.000	0.000	0.000
	(3)	1,026	1,025	1,022	988	734	835

(i) Frequency of contact with friends who are not neighbors; (ii) Family; (iii) Friends; (iv) Neighbors; (v) Partners; (vi) Professionals. (1) Pearson correlation. (2) Sig. (Bilateral). (3)

* marks that the correlation is significant at the 0.05 level

and

** marks that the correlation is significant at the 0.01 level.

#### Frequencies in carrying out activities and frequency of contact

Delving into the possible relationships that could be established between the frequencies of activities (D_3.2) and the frequency of contact with different groups of people (D_2), we found significant relationships between the different groups of variables (detecting two large correlation groups). On the one hand, the frequency of contact with non-family relationships (friends and neighbors) maintains a significant correlation (*p* < 0.01) with most of the leisure activities and activities leading to consumerism (Table 7).

**Table 7:** Correlational significance between the groups of variables (I).

		**Frequency in**					
		**i**	**ii**	**iii**	**iv**	**v**	**vi**
Frequency of contact with friends who are not neighbors	(1)	0.177^**^	0.133^**^	−0.235^**^	−0.387^**^	−0.196^**^	−0.187^**^
	(2)	0.000	0.001	0.000	0.002	0.000	0.000
	(3)	582	600	460	64	765	766
Frequency of contact with neighbors	(1)	0.172^**^	0.128^**^	−0.276^**^	0.251	−0.119^**^	−0.183^**^
	(2)	0.000	0.002	0.000	0.058	0.001	0.000
	(3)	549	563	423	58	723	716

(i) Visiting and receiving visits; (ii) Have lunch or dinner off home; (iii) Go for tapas, drinks, or have an aperitif; (iv) Go dancing; (v) Go for a walk (accompanied); (vi) Talk on the phone with family and friends. (1) Pearson correlation. (2) Sig. (Bilateral). (3)

** marks that the correlation is significant at the 0.01 level.

The article "Lifestyles of Spanish elders from supervened SARS-CoV-2 variant onwards: A correlational research on life satisfaction and social-relational praxes" was published in 2022. Journal: Front Psychol.

Within the second correlational group (Table 8), it can be observed that the frequency of contact with family relationships (children and grandchildren) also correlates significantly (*p* < 0.01) with the more traditional activities carried out more individually (talking on the phone with family and friends, walking, computer communications [chat, email, video conferencing], and going to the library or reading club).

**Table 8:** Correlational significance between the groups of variables (II).

		**Frequency to**			
		**i**	**ii**	**iii**	**iv**
Frequency of contact with friends who are not neighbors	(1)	0.136^**^	0.197^**^	−0.210^**^	−0.521^**^
	(2)	0.002	0.000	0.001	0.000
	(3)	535	530	242	50
Frequency of contact with neighbors	(1)	–	0.090^*^	−0.204^**^	−0.340^**^
	(2)	–	0.020	0.001	0.007
	(3)	–	673	271	61

(i) Go for a walk; (ii) Talk on the phone with family and friends; (iii) Manage computer communications; (iv) Go to the library or reading club. (1) Pearson correlation. (2) Sig. (Bilateral). (3)

* marks that the correlation is significant at the 0.05 level

and

** marks that the correlation is significant at the 0.01 level.

In sum, it can be said that revealed correlations point to two differential relationships and lifestyles that strengthen the frequency of different activities and social relationships in the elder. Digging deeper into such an observed lifestyle's dichotomy, variance remains explained at 23.6% in the linear regression analysis, introducing as a *dependent* variable the frequency in relationships with friends and as an *independent* variable the main variables displaying significant correlations. Consequently, the result yields an adjusted *R*^2^ of 0.236 [23.6% of the variance explained (Table 9)].

**Table 9:** Fitted model (I).

**Model**	***R***	***R^2^***	***R${}_{adj}^{2}$***	**Std. error of the estimate**
1	0.630^a^	0.397	0.236	0.71046

a Explanation of the regression model; Frequency of having lunch or dinner away from home; Frequency of visiting and receiving visitors; Frequency of talking on the phone with family and friends; Frequency of going dancing.

The article "Lifestyles of Spanish elders from supervened SARS-CoV-2 variant onwards: A correlational research on life satisfaction and social-relational praxes" was published in 2022. Journal: Front Psychol.

To what happens in the Fitted model (I), if we set the frequency of contact with offspring living outside locality boundaries, the *dependent* variable, and the group of variables with the highest correlation as the *independent* variable, the linear regression analysis provides a result of the model to an adjusted *R*^2^ of 0.451 [45.1% of the variance explained on the frequency of contact with offspring (Table 10)].

**Table 10:** Fitted model (II).

**Model**	***R***	***R^2^***	***R${}_{adj}^{2}$***	**Std. error of the estimate**
1	0.710^a^	0.504	0.451	0.70446

a Explanation of the regression model; Frequency of computer communications (chat, email, videoconferences); Frequency of going to the library, reading club; Frequency of talking on the phone with family and friends.

## Discussion

The original research goal and the three scrutinized dimensions revealed through the analysis that personal relationships still constitute themselves as the aspects of life displaying the highest satisfaction levels to those aged 65 and above residing in Castile-La Mancha, with family interaction being the most frequent of them all (every/almost every day). Such an aspect is initially worth to be mentioned because, despite the respiratory issues provoked by the SARS-CoV-2 retrovirus, the 40,000,000 diagnosed cases and the exceeding 1,100,000 deaths by 2020, and the social distancing and confinement or shelter-in-place measures (Palialol et al., 2020), the social relations prevail over other supposed essential aspects like health, self-skills, or wealth to the elders. So much so is this phenomenon that the high level of relational satisfaction with family and friends shows, at all times, a high correlation with satisfaction levels with the rest of the daily aspects of life. In this regard, there is coincident research pointing out the importance of social relationships in satisfaction with life and wellbeing (Cornwell et al., 2008; Litwin and Shiovitz-Ezra, 2011; Molero and Pérez-Fuentes, 2011; Pérez-Escoda, 2013; Rafnsson et al., 2015; Tomini et al., 2016; Burholt et al., 2020; LaBorde and Williams, 2022). However, in other studies, the time spent in social relationships reveals no correlation with life satisfaction (Triadó et al., 2009).

Despite the frequency of contact, the relationships with family scores as the most frequent, and to a lesser extent the socialization with friends or neighbors, those polled showing a high frequency of contact with any of these groups (family, friends, and neighbors) also revealed a high frequency with the other variables from the set. In this sense, although the adopted social distancing policies and measures were (and indeed still are) beneficial to stopping the spread out of the SARS-CoV-2 infection and saving lives (Thunström et al., 2020), we observed the use of alternative ways of interaction, i.e., in the study, a strong relationship between the variables “talking on the phone with relatives and friends” and “computer communications” (chat, email, video conferencing) with the variable “frequency of family relationships” was observed. From this particular piece of information, we can infer that, regardless of the social situation of each moment, there are interactional or socializing factors remaining constant or unaltered (even reinforced).

The article "Lifestyles of Spanish elders from supervened SARS-CoV-2 variant onwards: A correlational research on life satisfaction and social-relational praxes" was published in 2022. Journal: Front Psychol.

The above-referenced observation leads to deepening into the interactional differences revealed by participants. That is to say, those polled displaying higher punctuations in the frequency of contact with the “non-relatives” item conveyed an activity more related to *consumerism* and *leisureliness*. This result of leisure activities is coincident with Toepoel's (2013) research, which revealed greater social integration by the people connected to this variable. The post-pandemic scenario would represent a problem for this population because these activities tend to occur outside the home and in indoor locations (shopping centers, bars, restaurants, etc). Concerning this tendency, various studies proved the influence of both social relationships and activity and leisure on satisfaction with life in general (Cheng et al., 2009; Molero and Pérez-Fuentes, 2011; Li et al., 2021; Chen et al., 2022; Geithner and Wagner, 2022), as well as the connection between the performance of leisure activities and an increase in social connectivity (Toepoel, 2013), but the present research has just focused the attention on the interrelation between participant's relationships and the activities carried out. Outdoor activities do also imply significant cultural differences (Silverstein and Parker, 2002; Lee et al., 2014). Diametrically opposed, in our research, it was found that those polled manifesting higher contact frequency with “relatives” or “family” members correlated with the more *traditional* activities.

The differentiation of activities shown in the previous paragraph leads to the different lifestyles observed in participants. Previously, it was mentioned that, regarding the main activities of daily life, there was a group with a high correlation between the more traditional activities and a lower level of activity and another group with a correlation between activities more linked to consumption outside the home and more significant social activity. These dualities were kept when the three dimensions were analyzed two-by-two. For example, regarding the relationship between satisfaction levels and the frequency of contact with relationships, it was observed that personal contact increased satisfaction with life. Similarly, it was detected that the satisfaction level with the family was closely connected to the frequency of contact with family relationships (mainly children and grandchildren), while the satisfaction level with friends arises, to a greater extent, from the frequency of contact with friends and neighbors.

The article "Lifestyles of Spanish elders from supervened SARS-CoV-2 variant onwards: A correlational research on life satisfaction and social-relational praxes" was published in 2022. Journal: Front Psychol.

Regarding the connection between social relationships and satisfaction levels, other studies coincided with the present research (Fagerström et al., 2007; Triadó et al., 2009; Toepoel, 2013; Rafnsson et al., 2015; Steptoe and Fancourt, 2019). Two correlation groups showed two differentiated lifestyles concerning the relationship between frequency of contact and the activities carried out. That is, the frequency of contact with non-family relationships (friends and neighbors) maintained a strong influence on a large part of the leisure and consumption activities, while, in the second correlational group, it was observed that the frequency of contact with family relationships manifested a more substantial influence on the more traditional and solo activities.

In addition to the relationships found, other factors regarding this line of research could be investigated, which could be considered limitations in this study field, such as nutrition and physical activity. The relationship between physical activity and active and healthy aging is yet agreed upon. However, scientific evidence warns of the risks of physical activity that require significant effort. What has been pointed out is essential because 7.5% of the elderly in Castile-La Mancha who would carry out tasks that require great physical effort would be affected. Also, Vancini et al. (2021) showed that high-volume physical exercise with moments of maximum intensity, in the long term, is associated with an increased risk of myocardial infarction and other serious health problems. Regarding nutrition, although it is not part of this research, it could be interesting to incorporate the relationship between ingested food and fine motor and cognitive function. Concerning future and necessary research, Akbari et al. (2021) dug into an exciting topic in the field as the specific intake of certain micronutrients in a healthy diet and proved its correlation with *cognitive* performance and the level of physical activity in older adults.

The article "Lifestyles of Spanish elders from supervened SARS-CoV-2 variant onwards: A correlational research on life satisfaction and social-relational praxes" was published in 2022. Journal: Front Psychol.

## Conclusion

In sum, this study's contribution to science confirms the family's value for those aged 65 years and above and how they, far from substantially altering their life habits in the face of adversity, tend toward new forms of socialization and maintenance of leisure activities. In other words, social relations in the post-pandemic scenario remain as before the appearance of the virus and reappear with more force. Such relationships are constituted as the motor of both the satisfaction level with life and the diversity and frequency of daily life activities.

Although the previous aspect is general and applies to the entire population analyzed, there are two main lifestyles linked to the frequency and type of social relationships that occurred: one of a more traditional nature and linked to a high frequency in family relationships causing activities more traditional and with less social interaction and another with greater relevance and frequency in the relationships with non-family causing leisure activities, consumerism, and more significant social and relational activity.

In our view, such lifestyles should not be interpreted as exclusive but as intrinsic and underlying aspects of the elders' diversity, beliefs, and values. Regarding future research and shortcomings detected in the study, a larger-scale investigation incorporating participants from other cultures would have added additional value. In this sense, more studies would be necessary to verify the results in other countries and communities or cultures.

## Data availability statement

The raw data supporting the conclusions of this article will be made available by the authors. Requests to access the datasets have to be directed to the corresponding author.

## Author contributions

OD and PF: research design and data collection. IH: statistical analysis. JG: writing. All authors contributed to the article and approved the submitted version.

## Funding

This article is a by-product of a broader study entitled “Nuevos perfiles de la población mayor en Castilla-La Mancha”, a result of the collaboration between the European Network for the Fight against Poverty in Castilla-La Mancha (EAPN) and the University of Castilla-La Mancha (UCLM) from the core project SBPLY/19/270802/000377 named “Impulso y desarrollo de acciones de voluntariado en el marco de Envejecimiento Activo de los Centros de Mayores” and financed by the Regional Ministry of Social Welfare in Castilla-La Mancha, Spain.

## Conflict of interest

The authors declare that the research was conducted in the absence of any commercial or financial relationships that could be construed as a potential conflict of interest.

The article "Lifestyles of Spanish elders from supervened SARS-CoV-2 variant onwards: A correlational research on life satisfaction and social-relational praxes" was published in 2022. Journal: Front Psychol.

## Publisher's note

All claims expressed in this article are solely those of the authors and do not necessarily represent those of their affiliated organizations, or those of the publisher, the editors and the reviewers. Any product that may be evaluated in this article, or claim that may be made by its manufacturer, is not guaranteed or endorsed by the publisher.
